# Application of Refined Nursing Combined with Comprehensive Treatment of Traditional Chinese and Western Medicine in Gastrointestinal Dysfunction after Tumor Operation

**DOI:** 10.1155/2022/4957061

**Published:** 2022-07-20

**Authors:** Hongqing Su, Yuexian Wen, Dandan Kang

**Affiliations:** ^1^Traditional Chinese Medicine Department, Zhongshan Hospital Xiamen University, Xiamen 361004, China; ^2^Department of Gastrointestinal Surgery, Zhongshan Hospital Xiamen University, Xiamen361004, China

## Abstract

After surgical treatment, the gastrointestinal function of tumor patients is inhibited for a short time. Refined nursing is beneficial to the recovery of gastrointestinal function of tumor patients after operation. Traditional Chinese medicine and Western medicine have their own advantages in the treatment of gastrointestinal dysfunction after tumor operation and the combined application of the two is more ideal. Therefore, on the premise of refined nursing, we should carefully study the efficacy of integrated traditional Chinese and Western medicine in the treatment of postoperative gastrointestinal dysfunction in tumor patients. Fifty patients with gastrointestinal dysfunction after tumor surgery admitted to Xiamen University Affiliated Zhongshan Hospital from June 2021 to August 2022 were retrospectively selected. Twenty two of them received refined care + Western medicine (control group, CG) and the other 28 received refined care + Western medicine + moxibustion and thumb-tack needle Chinese medicine (observation group, OG). We compared the recovery of gastrointestinal function, inflammatory factors, negative emotions, sleep quality, length of stay, medical expenses, and adverse reactions. The postoperative recovery effect of gastrointestinal function in the OG was better than that in the CG. The IL-8 level and TNF -*α* level in OG were lower than those in CG. Relative to CG, the OG had significantly low SDS scores, SAS scores, PSQ1 scores, length of hospital stay, and medical expenses. The OG incidence of adverse reactions was 28.57%; it was significantly lower than 59.09% in the CG. Refined nursing with integrated Chinese and Western medicine therapeutic interventions can promote the recovery of gastrointestinal tract function, relieve anxiety and depression, and improve sleep quality in patients with postoperative gastrointestinal dysfunction after tumor surgery.

## 1. Introduction

Gastrointestinal dysfunction is a series of syndromes caused by short-term suppression of gastrointestinal function after clinical surgery [1], with the main clinical manifestations being diminished or absent bowel sounds, poor venting and defecation or even complete cessation, accompanied by abdominal distension, nausea, poor appetite, constipation, and fatigue. Therefore, the adoption of reasonable and effective nursing and therapeutic interventions to promote the recovery of the gastrointestinal function in postoperative patients has been a topic of great interest to health care professionals [2, 3]. Refined nursing care is based on the conventional nursing procedures and each procedure is then detailed. Moreover, the details are further optimized to make the entire nursing procedure more detailed and optimized. The better the nursing services the patients receive, the more confident they are in the recovery of the disease [4, 5].

At present, the clinical intervention methods include the use of drugs to promote gastrointestinal creep, gastrointestinal decompression, and other methods to promote the recovery of gastrointestinal dysfunction after abdominal surgery. However, factors such as postoperative fasting and stay on the bed can affect the recovery of gastrointestinal function. Moxibustion, as a commonly used traditional Chinese medicine therapy, has a wide range of adaptation, clinical indications in all branches, and is simple, easy to learn, and timely. Moxibustion therapy is not only used in hospitals but also can be used in families for self-therapy and mutual therapy, which is attached to the medical viewpoint of “early treatment is the most important” of Traditional Chinese medicine [6–8]. Moxibustion combines the properties of moxa leaves to promote the flow of Qi blood, warm the middle, and expel cold with the warm stimulation of moxibustion fire, which has the effect of warming the meridians, promoting the movement of Qi blood and the transportation of water and fluids [9, 10]. Therefore, it can effectively relieve postoperative abdominal pain, abdominal distension, and other symptoms. As a branch of acupuncture and moxibustion of Traditional Chinese medicine, the screw acupuncture treatment is the development and innovation of traditional intradermal acupuncture treatment. Clinically. we found that the duration of short-term inhibition of gastrointestinal function was different for each tumor patient after surgery. Therefore, it can stimulate the immune function of the body, reduce the sense of pain, and relieve gastrointestinal discomfort through long-time intradermal needle retention.

Traditional Chinese medicine and Western medicine have their own uniqueness to treat postoperative gastrointestinal dysfunction and the combined application of the two is more ideal. However, few studies have focused on the effect of fine nursing combined with integrated traditional Chinese and Western medicine on postoperative gastrointestinal function of tumor patients. This study retrospectively analyzed the clinical data of tumor patients who underwent surgical treatment, to investigate the effects of postoperative implementation of refined nursing combined with combined Chinese and Western medicine on gastrointestinal function of tumor patients and in order to provide a feasible intervention plan for the recovery of gastrointestinal function of tumor patients after surgery.

## 2. Cases and Methods

### 2.1. Cases

Fifty patients with gastrointestinal dysfunction after tumor surgery admitted to Xiamen University Affiliated Zhongshan Hospital from June 2021 to August 2022 were retrospectively selected. This study was conducted with the approval of the Ethics Committee.

#### 2.1.1. Inclusion Criteria

Tumor patients with surgical indications were confirmed by pathological biopsy, and tumor focus resection was successfully completed. The patients were between the age of 20 and 60 years. Two or more of the following symptoms after surgery, that is, after the removal of the gastric tube and after eating persistent abdominal distention, abdominal pain, repeated nausea, vomiting, vomiting symptoms relief, and delayed exhaust, defecation, tenesmus, etc. The duration of anesthesia is more than 2 hours. Patients are willing to participate and can actively cooperate.

#### 2.1.2. Exclusion Criteria

The patient had intestinal dysfunction or underwent intestinal surgery. The patient had anxiety, depression, or other mental disorders before surgery. Patients' own diseases that affect gastrointestinal dynamics, such as moderate or severe anemia, thyroid disease, and severe postoperative hypoproteinemia. The patient is allergic to medication.

22 cases received fine nursing + Western medicine and were set up as the control group (CG). The remaining 28 received fine care + Western medicine + Chinese medicine and were set up as an observation group (OG). The schematic diagram of the study is shown in Figure 1.

### 2.2. Methods

#### 2.2.1. In the CG

1. Psychological counseling: We made a preliminary assessment of the patient's psychological condition based on the actual condition of the patient, organ function, physical condition, medical history, and medication history, etc. Then, we looked for tendencies and problems that might affect the patient's mood, guided the patient to confide in his worries and doubts, and took psychological care measures to alleviate his fears in response to his psychological problems.
2. Patients were given a basic adjuvant therapy such as water fasting, oxygen, routine rehydration, anti-inflammatory, and total parenteral nutritional support.
3. We gently changed the dressing process for the patient and entrusted that patients with difficult defecation should not be forced to defecate, so as not to cause serious complications caused by blood vessel rupture. We let the patient watch their favorite TV series and read books to divert attention, relieve pain, when necessary, according to the doctor's advice to give analgesic drugs.
4. Privacy refinement care: Because of the special location of colorectal cancer surgery, some patients are concerned about exposing their private parts during the nursing operation, so we explain the purpose of the nursing operation to them in advance. Then, we used screens to shield the opposite sex temporarily and fully respect the privacy of patients.
5. If the patient's vital signs were stable 24 h after surgery, the next day, patients could turn in bed every 2 h and actively move the ankle joint of the lower limbs. We assisted the patient in a sitting position by elevating the head of the bed and adapted the patient to a sitting position as soon as possible and attempted to get out of bed after surgery.

#### 2.2.2. In the OG

On the basis of the CG, moxibustion and thumb-tack needle were performed.

Before moxibustion intervention, we informed patients of the moxibustion process and matters needing attention, combined with the principle of moxibustion, and emphasized the role of moxibustion in postoperative gastrointestinal function recovery. The specific steps are as follows: The patient lies flat and fully exposes the Shenque, Tianshu, Guanyuan, and Zusanli acupoints. The Shenque acupoint is located in the middle of the umbilicus. The Tianshu acupoint is located 2 inches away from horizontal umbilical midline. The Guanyuan acupoint is located in the anterior midline of the abdomen, 3 inches in the middle and lower umbilicus. The Zusanli acupoint is located in the anterolateral leg, a horizontal finger away from the tibial front. Moxibustion treatment is carried out from 7 : 00 to 9 : 00 every morning. Ignite moxa wick at about 1 horizontal finger away from the acupoint to ensure that the body surface temperature of the moxibustion point is about 45°C. Moxibustion is applied once a day for 30 minutes until the patient is exhausted after surgery. We will stop the moxibustion immediately if the patient experiences headache, nausea, and other adverse reactions during the moxibustion process. After the moxibustion is finished, we advise the patient to wash the local skin with warm water and keep warm.

The specifications for the operation of thumb-tack needle: The thumb-tack needle is 0.2 mm × 0.3 mm size for ear acupoints, including Shenmen, Trijiao, large intestine, small intestine, and stomach acupoint. Embedding method: We disinfect the skin with 75% alcohol, then place the thumb-tack needle on the corresponding point, and finally press vertically with the thumb or index finger. The technique is light to heavy, to produce a soreness and swelling. Pressing time: we press each point in turn for a total of 1 to 2 min each time, 3 times a day (08 : 00 : 00, 12 : 00 : 00, 18 : 00 : 00), by the responsible nurse on duty until the patient's gastrointestinal function is restored. Matters needing attention: The needle is left for 24 hours to replace. Timely replacement of tape edges if they buckle to ensure consistency of the needled area each time. Gentle movements when pressing the auricular points, it is appropriate for the patient to be painless to prevent auricular chondromalacia.

### 2.3. Observation of the Curative Effect

1. The first postoperative anal exhaust, time to first anal discharge, time to first postoperative bowel movement, time to recovery of bowel sounds, and time to bed activity were compared between the two groups. Bowel sound recovery time means hepatobiliary surgeon auscultated the patient's abdomen in four regions, upper right, lower right, upper left, and lower left, at intervals of 2 to 3 h for at least 1 min. Bowel sounds were detected more than 3 times/hour in ≥2 regions, and the recovery of bowel sounds was determined.
2. Peripheral venous blood was collected in the morning on an empty stomach one day before and 2 weeks after treatment, and the serum was routinely centrifuged to determine serum interleukin (IL)-8 and tumor necrosis factor (TNF)-*α* levels by ELISA.
3. The scores of anxiety and depression were observed. Self-rating Depression Scale (SDS) and Self-rating Anxiety Scale (SAS) [11] were used to score patients' depression and anxiety before and after treatment. The aggregate scores of SDS scale and SAS scale were 100 points, if the score is high, the patient's anxiety and depression become more grievous.
4. The Pittsburgh Sleep Quality Index (PSQ1) scale [12] was used to assess patients' sleep quality. The items involved in the scoring can be combined into 7 components, and each component is scored on a four-point scale from 0 to 3. The aggregate score is obtained by adding the scores of the seven parts. If the score is very high, it indicates that the sleep quality is poor.
5. Compared the two groups' length of hospital stay, medical expenses, and the incidence of adverse reactions, such as headache, nausea and vomiting, intradermal needle-related infection, tingling, and discomfort.

### 2.4. Statistical Analysis

SPSS 23.0 statistical software package was used for statistical analysis. The quantitative data were described in the form of mean and standard deviation (*M* ± SD). Categorical data were described using the number of cases (percentage). Chi-square test or ANOVA was used for analysis. *P* < 0.05 means the difference is statistically significant.

## 3. Results

### 3.1. Baseline Data

Most of the 50 patients were male, accounting for 62.0%, 72.0% lived in rural areas, and 38.0% had gastric cancer. There were no differences between the two groups in gender, age, BMI, education level, place of residence, disease type, and family history (*P* > 0.05) as shown in Table 1.

### 3.2. Comparison of Gastrointestinal Function Recovery between the Two Groups of Patients with Gastrointestinal Dysfunction

The postoperative recovery effect of gastrointestinal function was better in the OG, the first anal exhaust time was 16.35 h, the first postoperative defecation time was 29.65 h, the recovery time of bowel sound was 13.21 h, and the ambulation time was 14.25 h was significantly shorter than that of the CG as shown in Table 2.

### 3.3. Comparison of Inflammatory Factors between the Two Groups of Patients with Gastrointestinal Dysfunction after Tumor Surgery

After treatment, the levels of IL-8 and TNF -*α* in both groups were decreased. The levels of IL-8 and TNF -*α* in the OG after treatment were 30.65 ng/L and 15.74 pg/L, respectively. The levels of IL-8 and TNF -*α* in the control group were 40.65 ng/L and 21.09 pg/L, respectively. The OG was significantly lower than the CG as shown in Table 3.

### 3.4. Comparison of Negative Emotions between the Two Groups of Patients with Gastrointestinal Dysfunction after Tumor Surgery before and after Treatment

After treatment, SAS and SDS scores of the two groups decreased. SDS and SAS scores of the OG after treatment were 37.21 and 35.11, respectively. SDS and SAS scores of the CG were 47.18 and 47.36, respectively. Moreover, the OG was significantly lower than the CG as shown in Table 4 and Figure 2.

### 3.5. Comparison of Sleep Quality between the Two Groups of Patients with Gastrointestinal Dysfunction after Tumor Surgery before and after Treatment

After treatment, the PSQ1 score of the two groups decreased, and 8.39 in the OG was significantly lower than 10.82 in the CG as shown in Table 5.

### 3.6. Comparison of Hospitalization Time and Medical Expenses between the Two Groups of Patients with Gastrointestinal Dysfunction after Tumor Surgery

In terms of hospital stay and medical expenses, the OG value (9.17 days and 16,700 RNB) was significantly lower than the CG (13.05 days and 25,800 RNB, respectively) as shown in Table 6.

### 3.7. Comparison of the Incidence of Adverse Reactions between the Two Groups of Patients with Gastrointestinal Dysfunction after Tumor Surgery

There were 15 cases of adverse reactions in CG, with an incidence of 59.09%. There were 8 cases of adverse reactions in the OG, with an incidence of 28.57%. The incidence of adverse reactions in OG was significantly lower than that in CG.

## 4. Discussion

In the treatment of cancer diseases, surgical excision is indeed superior. However, due to various factors such as more complex diseases, preoperative anesthesia, intraoperative instrument pulling, and prolonged postoperative fasting, some patients have poor compliance and are prone to postoperative stress reactions [13]. Patients are prone to anxiety, panic, nausea and vomiting, abdominal distension and fullness discomfort, difficulty in venting and defecation, as well as intestinal adhesions, intestinal obstruction, abdominal masses, and other gastrointestinal autonomic paralysis and gastrointestinal dysfunction phenomena, which directly affect postoperative recovery and increase patients' anxiety. Therefore, nursing and treatment of cancer patients with poor compliance, postoperative stress response, anxiety, panic, gastrointestinal dysfunction, and other problems has still been the focus of clinical attention [2, 3].

With the change of clinical medical model and nursing concept, people's requirements for nursing services are increasing [14], which requires nursing staff to give different nursing methods according to different diseases and different patients to maximize the improvement of diseases and shorten the hospitalization time in order to reduce the economic pressure of patients. Conventional nursing measures lack of integrity and individuality and have weak control over details [15]. Cao et al. [16] have reported that a high level of nursing for postoperative patients with gastric cancer can improve their negative psychological mood. Refined care is the refinement of traditional care and the implementation of refined nursing interventions for patients based on individual differences, psychological, physiological, and overall, in all aspects, aiming to promote wound healing and improve clinical symptoms [4, 5, 17, 18]. On the basis of detailed care, this study explores the combination of traditional Chinese and Western medicine treatment of the postoperative gastrointestinal dysfunction in patients with tumor. Moreover, the results showed that compared with the CG, treatment group effect better recovery of gastrointestinal function, for the time to first anal discharge, time to first postoperative bowel movement, time to recovery of bowel sounds, and time to bed activity is significantly less time. It indicates that integrated traditional Chinese and Western medicine treatment is beneficial to postoperative gastrointestinal function and disease recovery, which is similar to the results of Li et.al. [10]. Moxibustion can promote local blood circulation in the abdominal gastrointestinal tissues, stimulate the nerves of the gastrointestinal tract, accelerate the metabolism of the gastrointestinal tract, and thus increase the rhythm of gastrointestinal peristalsis. Thumb-tack needle by press can help to adjust gastrointestinal nutrition balance, reduce abdominal pressure, regulate visceral function and dredge viscera meridians, and promote the early recovery of gastrointestinal function of patients.

Surgical treatment is an invasive treatment that has a great impact on stress response and inflammatory factors, among which IL-8 and TNF-*α* are common inflammatory factors that can activate the chain reaction of inflammatory factors. It can improve the activity of phagocytes, increase the degree of inflammatory response, and aggravate gastrointestinal dysfunction [19]. Cho et.al. [20] showed that acupoint pairing enhances clinical effects and that correct and reasonable acupoint pairing is the key to the efficacy of acupoint stimulation. Therefore, this study selected Shenque, Tianshu, Guanyuan, Zusanli acupoints, and ear acupoints for moxibustion and thumb-tack needle treatment, showing that the levels of IL-8 and TNF-*α* in the OG were significantly lower than those in the CG, indicating that integrated traditional Chinese and Western medicine has a better effect on reducing the level of inflammatory factors in tumor patients, which is similar to the research results of Wang et.al. [21]. We evaluated the anxiety, depression, and sleep quality of the tumor patients before and after treatment, and the results showed that the SAS, SDS, and PSQ1 scores of the OG were lower than those of the CG. Wang et.al. [22] concluded that combined Chinese and Western medicine treatment of patients with severe community-acquired pneumonia can reduce treatment failure, time to clinical stabilization, length of hospitalization, and in-hospital mortality, and improve quality of life. Luo et.al. [23] found that based on “Biaoben acupoint compatibility”, thumb-tack needle could significantly reduce the sequelae symptoms, anxiety and depression, help patients adjust their mood, and improve sleep in patients recovering from neocon pneumonia disease. The results were similar to those of our study. Lv et al. [24] showed that acupuncture therapy, as a non-drug treatment for the prevention and treatment of nausea and vomiting in traditional Chinese medicine, has a definite curative effect. The thumb-tack needle is buried under the skin to produce continuous and stable stimulation, which facilitates the movement of Qi blood in the meridians. All the indications of acupuncture can be used with intradermal embedding acupuncture, which has little influence on patients' movement in the process of application and avoids the discomfort caused by single postures after surgery. The short thumb-tack needle body of the snap basically has no hidden danger after application [25]. The results showed that the length of hospital stay, medical expenses and incidence of adverse reactions in the OG were lower than those in the CG, indicating that fine nursing combined with traditional Chinese and Western medicine can improve the treatment effect, reduce the economic burden of patients in hospital, and alleviate the development of postoperative adverse events.

## 5. Strengths and Limitations

Integrated treatment with the Chinese and Western medicine theories is a new medical concept, which can further improve the prognosis of patients by implementing refined care along with the characteristic evidence-based treatment of Chinese medicine. However, the small sample size and short follow-up time of this study make its findings have some limitations. In the later clinical work, the sample size can be expanded and the study time extended to further evaluate the patients' treatment compliance and analyze the risk factors affecting their poor prognosis, etc. The above problems will continue to be added and studied gradually at a later stage.

## 6. Conclusions

Postoperative care and treatment for cancer patients are developing and improving. A retrospective analysis found that meticulous nursing combined with integrated traditional Chinese and western medicine has a significant effect on the treatment of gastrointestinal dysfunction after tumor surgery. It can promote the recovery of gastrointestinal function, reduce the level of inflammatory factors, relieve anxiety and depression, improve sleep quality, shorten hospitalization time, reduce costs, and improve treatment safety.

## Figures and Tables

**Figure 1:** The schematic diagram of the study.

**Figure 2:** (a) Comparison of SDS scores between the two groups of patients with gastrointestinal dysfunction after tumor surgery before and after treatment. (b) SAS score comparison between the two groups of patients with gastrointestinal dysfunction after tumor surgery before and after treatment.

**Table 1:** Baseline data [*n* (%), *M *±* *SD].

Data		CG (*n* = 22)	OG (*n* = 28)	*t/χ * ^2^ value	*P* value
Gender	Men	13	18	0.141	>0.05
	Women	9	10		

Age (years)		28∼54	29∼60	0.789	>0.05
		46.32 ± 8.53	44.25 ± 9.71		
BMI (kg/m^2^)		25.65 ± 6.26	25.75 ± 2.06	0.079	>0.05

Education level	Primary school and below	4	3	0.681	>0.05
	Middle school	5	7		
	High school	5	8		
	College degree or above	8	10		

Place of residence	City	6	8	0.010	>0.05
	Countryside	16	20		

Disease type	Stomach cancer	7	12	3.547	>0.05
	Colorectal cancer	1	3		
	Pancreatic cancer	6	4		
	Esophageal cancer	5	3		
	Primary liver cancer	3	6		

Family history	Yes	7	6	0.691	>0.05
	No	15	22		

Family history refers to the development of the disease in family members (a larger range of family members, not limited to immediate family members such as grandchildren) of patients with gastric, colorectal, pancreatic, esophageal, and primary liver cancers. Some patients have hypertension, diabetes, or other underlying diseases.

**Table 2:** Comparison of gastrointestinal function recovery time between the two groups (h, *M *±* *SD).

Group	*n*	Time to first anal discharge	Time to first postoperative bowel movement	Time to recovery of bowel sounds	Time to bed activity
CG	22	23.56 ± 7.04	40.58 ± 11.36	20.47 ± 6.98	25.12 ± 8.35
OG	28	16.35 ± 4.25	29.65 ± 6.99	13.21 ± 2.87	14.25 ± 3.36
*t* value		4.485	4.187	5.003	6.285
*P* value		<0.05	<0.05	<0.05	<0.05

**Table 3:** Comparison of inflammatory factors between the two groups before and after treatment.

Group	*n*	IL-8 (ng/L)		TNF-*α* (pg/L)	
		Before	After	Before	After
CG	22	85.31 ± 14.57	40.65 ± 6.98	30.06 ± 4.15	21.09 ± 4.68
OG	28	82.36 ± 12.54	30.65 ± 5.14	29.65 ± 4.12	15.74 ± 3.03
*t* value		0.769	5.836	0.348	4.890
*P* value		>0.05	<0.05	>0.05	<0.05

**Table 4:** Comparison of negative emotions between the two groups before and after treatment.

Group	*n*	SDS score		SAS score	
		Before	After	Before	After
CG	22	69.55 ± 10.32	47.18 ± 6.23	66.18 ± 8.04	47.36 ± 4.07
OG	28	70.04 ± 11.32	37.21 ± 4.23	68.21 ± 9.93	35.11 ± 5.69
*t* value		0.160	6.729	0.779	5.822
*P* value		>0.05	<0.05	>0.05	<0.05

**Table 5:** Comparison of sleep quality between the two groups before and after treatment.

Group	*n*	PSQ1 score	
		Before	After
CG	22	15.82 ± 2.87	10.82 ± 2.11
OG	28	16.64 ± 2.59	8.39 ± 1.17
*t* value		1.060	5.174
*P* Value		>0.05	<0.05

**Table 6:** Comparison of hospital stay and medical expenses between the two groups.

Group	*n*	Length of hospital stay (d)	Medical expenses (ten thousand yuan)
CG	22	13.05 ± 3.65	2.58 ± 0.34
OG	28	9.17 ± 1.68	1.67 ± 0.52
*t* value		5.040	7.095
*P* Value		<0.05	<0.05

## Data Availability

The data used to support the findings of this study are available from the corresponding author upon request.
